The article "Effects of 5.8 GHz Microwaves on Testicular Structure and Function in Rats" was published in 2022. Journal: Biomed Res Int.

# Effects of 5.8 GHz Microwaves on Testicular Structure and Function in Rats

**DOI:** 10.1155/2022/5182172

**Published:** 2022-06-06

**Authors:** Yizhe Xue, Ling Guo, Jiajin Lin, Panpan Lai, Gang Rui, Liyuan Liu, Rongrong Huang, Yuntao Jing, Fuli Wang, Guirong Ding

**Affiliations:** ^1^Department of Radiation Protection Medicine, School of Military Preventive Medicine, Air Force Medical University, Xi'an, China; ^2^Ministry of Education Key Lab of Hazard Assessment and Control in Special Operational Environment, Xi'an, China; ^3^Department of Urology, Xijing Hospital, Air Force Medical University, Xi'an, China

## Abstract

**Objective:**

To investigate the effects of exposure to 5.8 GHz microwaves on testicular structure and function of male adult rats.

**Methods:**

After 30 days of exposure, we evaluated sperm quality by determining sperm concentration and quantifying the number of abnormal sperm. Testicular morphology was investigated by hematoxylin-eosin (HE) staining. The levels of testosterone (T), follicle-stimulating hormone (FSH), luteinizing hormone (LH), glial cell line-derived neurotrophic factor (GDNF), stem cell factor (SCF), and transferrin (TRF) were determined by enzyme-linked immunosorbent assays (ELISAs). We also used western blotting to determine the levels of GDNF and SCF and apoptosis-related protein (caspase-3) in the testis.

**Results:**

Compared with the sham group, there were no significant differences in terms of sperm count, sperm abnormality, and the levels of T, FSH, LH, GDNF, SCF, and caspase-3 in the microwave group.

**Conclusion:**

Under the experimental conditions, 5.8 GHz microwave exposure has no obvious effect on testicular structure and function of rats.

## 1. Introduction

Microwaves is a form of electromagnetic radiation with frequencies in the range of 300 MHz to 300 GHz that is used predominantly for radar, satellite communication, and radio navigation. In an attempt to meet the increasing demand for technology in modern-day life, the communications industry continuously strives to build network environments with higher efficiency, faster connections, and lower latency. Over the last few years, there has been a rapid development in 5 G networks in China. As a result, innumerable 5 G base stations and antennas will be installed in every corner of the country. It is also evident that the 5.8 GHz spectrum is likely to replace the 2.4 GHz spectrum that is currently used in wireless technology. However, there are some concerns over whether these new technologies will have a potential adverse impact on human health.

A growing body of scientists has become aware of this problem and has begun to conduct studies *in vitro*. For example, Miyakoshi et al. showed that exposure to 5.8 GHz microwaves at 1 mW/cm^2^ for 24 h had little or no genetic toxicity to human eye cells [1]. In another study, Kuzniar et al. used proteome-wide semiquantitative mass spectrometry to demonstrate changes in the protein abundance of three cell types (human fibroblasts, osteosarcomas, and mouse embryonic stem cells) when exposed to 5.8 GHz microwaves [2].

Previous research has demonstrated that the testis is a target organ that is highly sensitive to microwave exposure. There is also limited evidence that microwave exposure may be associated with poor sperm quality [3–5]. Jong et al. previously demonstrated a reduction in sperm concentration in rats when exposed for 30 days to microwaves emitted from 4 G mobile phones, thus indicating that a long period of exposure to microwaves had a clear effect on spermatogenesis [3]. In another study, Shahin et al. reported that that exposure to 2.45 GHz microwaves for 2 h/day over 15, 30, and 60 days led to a reduction in sperm concentration and survival in mice; this was accompanied by a reduction in testosterone levels and an imbalance in testicular redox status [4, 5]. The specific effects of 5.8 GHz microwaves on testicular structure and function have yet to be reported. Therefore, the purpose of this study was to investigate the effects of 5.8 GHz microwaves on testicular structure and function in a rat model.

## 2. Materials and Methods

### 2.1. Animals

36 healthy adult male Sprague-Dawley (SD) rats (body weight: 180.35 ± 8.45 g) were purchased from the Laboratory Animal Center of Air Force Medical University (Xi'an, China) and maintained under strict hygienic and well-ventilated conditions (temperature, 23 ± 2°C; humidity, 50% ± 2%; and a 12 h light/dark) with free access to food and water. All animal experiments in this study were approved by the Animal Welfare Committee of Air Force Military Medical University (Xi'an, China).

### 2.2. Exposure and Groups

The rats were randomly divided into two groups: a microwave group and a sham group (*n* = 18 for each group). The exposure system consisted of a signal generator, an amplifier, and a radiating antenna. Details on the exposure method have been published in our previous article [6]. Briefly, the rats were exposed or sham-exposed separately to 5.8 GHz microwaves for 1 h/d for 30 consecutive days. The exposure of microwaves group was conducted from 8:00 to 12:00 AM. The power density was 74.25 W/m^2^, the whole-body specific absorption rate (SAR) was 1.15 W/kg, and the SAR for the testis was 3.36 W/kg, which were calculated using XFDTD software with a rat model (body mass: 307.8 g) provided by Remcom (State College, PA, USA). The power density and SAR decreased with increasing the distance from the center, and the maximum attenuation value was approximately 3 dB. The rats in the sham group were treated in the same way as the microwave group but with zero output from the exposure system. The rectal temperature of each rat was measured immediately before and after exposure to 5.8 GHz microwaves. Besides, we measured the weight of each rat in both groups every three days.

### 2.3. Blood Collection and Tissue Sampling

At the end of 30-day exposure to microwaves, all rats were anesthetized with 1% sodium pentobarbital (60 mg/kg). Blood samples were collected from the left ventricle of hearts of 13 rats in each group, subsequently centrifuged at 3000 rpm for 10 minutes at 4°C to provide serum for the analysis of sex hormones. The bilateral testes and cauda epididymides were isolated immediately and washed with precooled phosphate-buffered saline (PBS, pH 7.4). Sperms were then collected from the bilateral cauda epididymides and used to measure sperm quality. The testicular index was calculated by the following formula: bilateral testes weight (g)/body weight (g) × 100. The remaining 5 rats in each group were anesthetized as described above and then perfused (via the intracardiac route) with cold 0.9% sodium chloride and 4% paraformaldehyde (PFA). Finally, the testes were fixed in 4% PFA for routine histological examination.

### 2.4. Sperm Count and Abnormality Analysis

The bilateral cauda epididymides of each rat (*n* = 13 for each group) were gently cut and placed in a 12-well plate containing 1 ml of sperm culture medium (M2, Millipore, MA, USA) and shaken slowly on a shaker for 30 minutes. The epididymides were then incubated at 37°C for 20 minutes to generate a suspension of sperm. Sperm were counted using a method that was described previously [7]. A sample of sperm suspension was then smeared on a glass slide and air-dried, fixed with precooled acetone for 20 minutes, stained with 2% eosin for 30 minutes. Sperm morphology was then assessed with a light microscope (Leica, Heidelberg, Germany). Approximately 400 sperm cells were examined from different visual fields on each slide to determine abnormal morphology, including amorphous, hookless, bicephalic, coiled, or abnormal tails, as described previously [8].

### 2.5. Testicular Histology

After fixation for 24 h, the testes were trimmed, dehydrated, cleared, dipped in wax, embedded in paraffin, and then sectioned serially with a rotary microtome (LeicaRM2135, Heidelberg, Germany) at a thickness of 5 *μ*m. Sections were then stained with hematoxylin-eosin (HE) under conventional procedures. A light microscope (Leica, Heidelberg, Germany) was then used to observe testicular morphology.

### 2.6. Enzyme-Linked Immunosorbent Assay (ELISA)

Lysing testicular tissue (*n* = 5 for each group) with radio immunoprecipitation assay (RIPA) lysis buffer was supplemented with phenylmethanesulfonyl fluoride and phosphatase/protease inhibitors (KeyGEN Biotech, Nanjing, China). The testicular tissue was then homogenized (12000 rpm for 10 min at 4°C) to extract total proteins with a homogenizer device (Leica). The levels of glial cell line-derived neurotrophic factor (GDNF), stem cell factor (SCF), and transferrin (TRF) in testicular tissue were then determined by commercial enzyme-linked immunosorbent assay (ELISA) kits (ML Bio, Shanghai, China) following the manufacturer's instructions. Besides, the serum levels of sex hormones (*n* = 5 for each group), including testosterone (T), follicle-stimulating hormone (FSH), and luteinizing hormone (LH), were also determined by ELISA kits (ML Bio).

### 2.7. Western Blotting

First, we determined the concentration of total protein in each sample (*n* = 5 for each group) using a Bicinchoninic Acid Protein Assay Kit (Beyotime, Shanghai, China). 10% sodium dodecyl sulfate-polyacrylamide gel electrophoresis (SDS-PAGE) was used to separate 30 *μ*g of protein from each sample. Then, the protein was transferred onto polyvinylidene fluoride (PVDF) membranes (Millipore, MA, USA). Membranes were then blocked with 5% nonfat milk for 2 h at room temperature and incubated with primary antibody overnight at 4°C using the dilutions listed in Table 1. After being rewarmed, the membranes were then incubated with species-matched horseradish peroxidase- (HRP-) conjugated secondary antibody (1 : 5000, CWBIO, Beijing, China) for 2 h at room temperature. Then, the protein signals were developed using the Universal Hood II Electrophoresis Imaging Cabinet (Bio-Rad, Milan, Italy). Immunoreactive bands were then quantified using Quantity One 4.62 software (Bio-Rad).

### 2.8. Statistical Analysis

All data were presented as the mean ± standard deviation (SD) and analyzed by two-tailed, Student's *t*-tests using SPSS version 20.0 software (SPSS Inc., Chicago, IL, USA) GraphPad Prism version 5.04 software (San Diego, CA, USA) was used to generate figures and graphs. Besides, all subjective analyses were performed by the individual blinded to group of exposure. *P* < 0.05 was considered to be statistically significant.

## 3. Results

### 3.1. Effects of Exposure to 5.8 GHz Microwaves on General Body Condition

As shown in Figure 1(a), 5.8 GHz microwave exposure caused an increase in rectal temperature of <1°C in rats. After 30 days of continuous exposure to 5.8 GHz microwaves, it was evident that the rats in each group had gained weight. There were no significant differences between the sham group and the microwave group in terms of body weight growth curve (Figure 1(b)), testicular weight (Figure 1(c)), and testis index (Figure 1(d)) (*P* > 0.05). These results indicated that exposure to 5.8 GHz microwaves had no significant effect on the general body condition of rats.

### 3.2. Effects of Exposure to 5.8 GHz Microwaves on Sperm Count and Abnormality

After 30 days of continuous exposure to 5.8 GHz microwaves, there were no significant differences between the sham group and the microwave group with regard to sperm count (Figure 2(a)) and the proportion of abnormal sperm (Figure 2(b)) (*P* > 0.05). These results indicated that exposure to 5.8 GHz microwaves under our experimental conditions had no significant effect on sperm count and abnormality in rats.

### 3.3. Effects of Exposure to 5.8 GHz Microwaves on Testicular Histological Structure

Figure 3 showed representative images of testicular morphology. There were no obvious differences between the sham and microwave groups with regard to testicular histology. The basement membrane of the spermatogenic epithelium was intact in both groups. Furthermore, the structure of the spermatogenic tubules and interstitial tissue was normal. There were innumerable mature sperm in the lumen, and spermatogenic cells at all stages of development were neatly arranged in layers around the lumen of the tubules.

### 3.4. Effects of Exposure to 5.8 GHz Microwaves on Serum Levels of Sex Hormones

As shown in Figure 4, after 30 days of exposure to 5.8 GHz microwaves, there were no significant differences between the sham group and the microwave group in terms of the serum levels of FSH, LH, or T (*P* > 0.05). These results indicated that exposure to 5.8 GHz microwaves for 30 days had no significant effect on the serum levels of sex hormones detected above.

### 3.5. Effects of Exposure to 5.8 GHz Microwaves on Testicular Secretory Function

As shown in Figure 5, after 30 days of exposure to 5.8 GHz microwaves, there were no significant differences between the sham group and the microwave group in terms of the serum levels of factors secreted from the Sertoli cells, including GDNF, SCF, and TRF (*P* > 0.05); this was the case for both ELISA results (Figures 5(a)–5(c)) and western blotting results (Figures 5(d)–5(f)). These results indicated that under our experimental conditions, exposure to 5.8 GHz microwaves for 30 days did not affect the secretory function of Sertoli cells.

### 3.6. Effects of Exposure to 5.8 GHz Microwaves on Testicular Cells Apoptosis

The expression levels of apoptosis-related protein (caspase-3) in testicular tissue were detected by western blotting. Caspase-3 is the most important terminal cleavage enzyme in the process of apoptosis. After 30 days of exposure to 5.8 GHz microwaves, there were no significant differences between the sham group and the microwave group in terms of the protein levels of caspase-3 in the testicular tissue (Figure 6) (*P* > 0.05). These results indicated that under these experimental conditions, exposure to 5.8 GHz microwaves for 30 days did not have any significant effect on apoptosis in testicular cells from rats.

## 4. Discussion

According to the previous Institute of Electrical and Electronics Engineers (IEEE) standards [9], the power density limit for occupational exposure at 5.8 GHz spectrum was set to 100 W/m^2^. However, this limit was adjusted to 50 W/m^2^ in the latest IEEE standards [10]. Given the evolving nature of the IEEE standards, we selected 75 W/m^2^ as the power density of microwaves to use in this study; the actual measured value was 74.25 W/m^2^. Under these conditions, the whole-body SAR of the experimental rats was 1.15 W/kg; this was lower than the threshold for thermal effects (4 W/kg). This was consistent with the fact that we observed no significant increase in the rectal temperature of experimental rats during this study.

It was reported an international action plan for the development of 5 G networks has begun and involves an increment in power density and using millimeter waves in the future [11]. Some reports have indicated that exposure to microwaves might cause a reduction in sperm count and vitality [4, 5, 7, 12] and cause damage to the morphology of testicular tissue [13]. However, some studies have reported the opposite result. For example, Imai et al. [14] exposed the whole bodies of rats to 1.95 GHz wideband code division multiple access signals (the freedom for mobile multimedia access strategy) for 5 h/day, 7 days/week for 5 weeks, and did not observe any significant changes in a range of indicators, including body weight, testicular weight, and sperm count. In another study, rats were exposed to 915 MHz radiation for 1 h/day for 2 weeks; no significant changes were detected with regard to testicular function and structure [15]. Therefore, there is a clear need to carry out a detailed investigation of the effects of microwave exposure on testicular structure and function in adult male rats. In the present study, we exposed rats to 5.8 GHz microwaves for 30 days and then investigated a range of indicators, including sperm count and abnormality, the secretory function of the Sertoli and Leydig cells, the morphology of testicular tissue, and the extent of apoptosis.

A previous study reported that long durations of exposure to an electromagnetic field led to a reduction in sperm count of SD rats [3]. Yan et al. [16] also reported that the exposure of rats to a 1.9 GHz radiation field generated by mobile telephone caused a significant reduction in sperm count and survival rate. In our experiment, the exposure of rats to 5.8 GHz microwaves for 30 days did not cause any significant changes in sperm count or the proportion of abnormal sperm, thus indicating that under our experimental conditions, exposure to 5.8 GHz microwaves had no significant effect on sperm count and abnormality. These findings are consistent with those previous reports [14, 17]. Further studies have focused on the effects of exposure to microwaves in living environments on sperm quality over the last few years. However, there is no definitive conclusion as yet.

Sertoli cells within the testicular tissue are known to provide nutrients for the development and reproduction of germ cells through secreting several important factors into the testicular environment, including GDNF, SCF, and TRF [18, 19]. They also maintain the balance of the microenvironment in spermatogenic tubules, thus playing a key role in spermatogenesis. GDNF promotes the proliferation of non-differentiated spermatogonia (including spermatogonial stem cells) [20] while SCF promotes the differentiation of spermatogonia into round sperm cells [21]. TRF is an objective indicator that reflects the secretory function of testicular Sertoli cells and is known to facilitate the transfer of iron from the serum to developing germ cells *via* the blood-testis barrier to maintain normal growth and maturation [22]. In our experiments, there was no significant difference between the sham group and the microwave group concerning the levels of GDNF, SCF, or TRF. These data indicated that under our experimental conditions, exposure to 5.8 GHz microwaves had no significant effect on the secretory function of the Sertoli cells in the testes of experimental rats. In addition, exposure to 5.8 GHz microwaves did not have any significant effect on body weight, testicular weight, or testicular morphology.

Testosterone is a steroid hormone that is mainly produced by the Leydig cells and induces the transformation of spermatocytes into sperm cells, thereby promoting the production and development of sperm cells and playing a key role in spermatogenesis [23]. FSH acts *via* receptors on the Sertoli cells to stimulate spermatogenesis, and LH induces Leydig cells to synthesize and secrete T [24]. In a previous experiment, 12-week-old male mice were exposed to 2.45 GHz microwaves (2 h/day for 30 days, power density = 0.029812 mW/cm^2^) and experienced a reduction in the serum levels of T [25]. However, many other studies have reported conflicting results. For example, the repeated exposure of mice to microwaves at 0.018-0.023 W/kg whole-body SAR led to an elevation of serum T; however, no histopathological alterations were detected in the reproductive organs [26]. In our experiments, we found no significant differences between the sham group and the group exposed to 5.8 GHz microwaves with regard to T, FSH, and LH. These differences between studies may be related to differences in animal strains, age, gender, and the microwave parameters applied, thus leading to conflicting results.

Some previous studies have shown that exposure to microwaves under certain conditions could induce apoptosis in the testicular cells [27, 28]. However, one previous study showed that exposure to 900 MHz radiation for 10 months (2 h/day, 7 days/week) did not affect the levels of cleaved-caspase-3 in the testes [29]. Similarly, we found that exposure to 5.8 GHz microwaves (1 h/day for 30 days) did not affect the levels of caspase-3 in the testes, which suggested that the canonical pathway of apoptosis was not activated after 5.8 GHz microwave exposure.

The results in this study indicated that exposure to 5.8 GHz microwave for 30 d has no obvious effects on the testicular function including spermatogenesis in rats. Since there is a big difference in histone organization and micro-RNA in the packaged sperm nuclei between rat and human, the conclusion drawn in this study cannot extend to human directly; unless, more epidemiological and experimental evidences are found in the future.

## 5. Conclusions

Under the experimental conditions used in the present study, 5.8 GHz microwaves did not induce any testicular structure damage and endocrine disruption of rats. Whether a longer exposure time or increased exposure intensities will result in damage has yet to be elucidated. The rat model is not fully representative of the human body. We hope more researchers pay attention to the effects of electromagnetic radiation produced by 5 G communication on the human body, and more epidemiological data will be available to support this study.

## Figures and Tables

**Figure 1:** Effects of exposure to 5.8 GHz microwaves on the general body condition of SD rats. (a) Change of rectal temperature. (b) Growth curve of body weight; *N* = 18 for each group. (c) Testis weight; *N* = 13 for each group. (d) Testis index (bilateral testes weight (g)/body weight (g) × 100). The values are expressed as the mean ± SD. *N* = 13 for each group.

**Figure 2:** Effects of exposure to 5.8 GHz microwaves on sperm quality of SD rats. (a) Sperm count. (b) Sperm abnormality. The values are expressed as the mean ± SD. *N* = 13 for each group.

**Figure 3:** Effects of exposure to 5.8 GHz microwaves on testicular morphology of SD rats. HE staining; *N* = 5 for each group; scale bar = 200 *μ*m or 100 *μ*m.

**Figure 4:** Effects of exposure to 5.8 GHz microwaves on the sex hormones of serum detected by ELISA. (a) FSH concentration. (b) LH concentration. (c) T concentration. The values are expressed as the mean ± SD. *N* = 5 for each group.

**Figure 5:** Effects of exposure to 5.8 GHz microwaves on the secreting function of testicular Sertoli cells in SD rats. (a–c) The ELISA results of the secreting function of testicular Sertoli cells. (a) GDNF. (b) SCF. (c) TRF. (d–f) The protein levels of GDNF and SCF in testicular tissue were measured by western blotting. (d) Typical immunoblots of GDNF and SCF. (e) Relative expression of GDNF. (f) Relative expression of SCF. The values are expressed as the mean ± SD. *N* = 5 for each group.

**Figure 6:** Effects of exposure to 5.8 GHz microwaves on the apoptosis-related protein in testicular tissue of SD rats detected by western blotting. (a) Typical immunoblots of caspase-3. (b) Relative expression of caspase-3. The values are expressed as the mean ± SD. *N* = 5 for each group.

**Table 1:** Antibodies used for western blotting.

Antibody	Species	Company	City and country	Dilution
Anti-*β*-actin	Mouse monoclonal Ab	CMCTAG	Milwaukee, WI, USA	1 : 5000
Anti-GDNF	Rabbit Polyclonal Ab	Abcam	Cambridge, England	1 : 400
Anti-SCF	Rabbit Polyclonal Ab	SAB	College Park, Maryland, USA	1 : 300
Anti-Caspase-3	Rabbit Polyclonal Ab	Proteintech	Wuhan, China	1 : 600

## Data Availability

The data are presented in the article.
